The article "DCE-DForest: A Deep Forest Model for the Prediction of Anticancer Drug Combination Effects" was published in 2022. Journal: Comput Math Methods Med.

# DCE-DForest: A Deep Forest Model for the Prediction of Anticancer Drug Combination Effects

**DOI:** 10.1155/2022/8693746

**Published:** 2022-06-09

**Authors:** Wei Zhang, Ziyun Xue, Zhong Li, Huichao Yin

**Affiliations:** ^1^Institute of Intelligent Emergency Information Processing, Institute of Disaster Prevention, Langfang 065201, China; ^2^School of Emergency Management, Institute of Disaster Prevention, Langfang 065201, China; ^3^School of Information Engineering, Institute of Disaster Prevention, Langfang 065201, China

## Abstract

Drug combinations have recently been studied intensively due to their critical role in cancer treatment. Computational prediction of drug synergy has become a popular alternative strategy to experimental methods for anticancer drug synergy predictions. In this paper, a deep learning model called DCE-DForest is proposed to predict the synergistic effect of drug combinations. To sufficiently extract drug information, the paper leverages BERT (Bidirectional Encoder Representations from Transformers) to encode the drug and the deep forest to model the nonlinear relationship between the drugs and cell lines. The experimental results on the synergy datasets demonstrate that the proposed method consistently shows superior performance over the other machine learning models.

## 1. Introduction

The traditional treatment mode of “single disease, single drug, and single target” faces the challenges of complex diseases, such as drug resistance, cancer recurrence, low response rate, and adverse side effects. To overcome the limitations of monotherapy, combination therapy is a promising treatment strategy. In combination therapy, a variety of drugs can target multiple targets and pathways, which can improve the therapeutic effect. At present, drug combinations are increasingly used to treat various complex diseases, such as hypertension, infectious diseases, and cancer. However, currently, there are more than 200 types of cancer chemotherapy drugs certified by the FDA, and the combination of random pairings between these drugs is as high as 19900. Relying on traditional experimental methods to screen the combination of synergistic antitumor drugs is very challenging in terms of time, efficiency, and cost. Therefore, there is an urgent need for computational methods to reduce the screening space of drug combinations. In the past few years, computational methods have been widely used in the prediction of drug combinations.

In recent years, several large-scale high-quality drug combination datasets have been released to support the rapid development of computational assisted drug combination screening. The computational methods can be classified into five categories: system biology methods, mathematical methods, stochastic search algorithms, kinetic models, and machine learning (ML) methods. The first four methods are based on hypothesis-driven computational methods, which are limited by the a priori knowledge. The ML-based methods can learn the complex nonlinear relationships between the input features and the output label. ML-based methods have been successfully applied to the field of drug combination, such as the gradient tree boosting classifier [1], support vector machine (SVM), and extreme gradient boosting (XGBoost). These classical ML methods need to rely on handcrafted features, which also depends on the professional knowledge.

The article "DCE-DForest: A Deep Forest Model for the Prediction of Anticancer Drug Combination Effects" was published in 2022. Journal: Comput Math Methods Med.

Recently, deep learning algorithms provide another path for drug development and invention that does not need to rely too much on handcrafted features. For example, DeepSynergy combined the chemical descriptors of drugs and gene expression of cell lines to predict the drug synergies based on three-layer feed-forward neural network [2]. Xia et al. proposed a novel deep learning model for the drug combination screening that integrates information from gene expression, microRNA expression, protein abundance, and 30 categories of molecular descriptors [3]. TranSynergy considered the network information such as gene-gene interaction networks and drug-target associations and applied the attention mechanism to improve the performance of deep learning model [4]. Different from the previous deep learning model, AuDNNsynergy first applied the Autoencoder to encode new vector representations for chemical structure of drugs and multiomics data of cell lines and then used the encoded features as final representation of drug and cell line [5]. DeepDDS applied the graph neural network (GNN) to learn the drug representation from the chemical structure [6].

In this paper, a novel approach that combined deep forest with BERT embedding for drug [7] for drug synergy prediction is proposed. It is designed to predict the drug synergy directly from the compound SMILES and gene expression. With the experimental dataset of drug synergy prediction, the DCE-DForest significantly outperformed the classical machine learning methods and other deep learning models.

## 2. Materials and Methods

### 2.1. About Datasets

In the experiment, authors use the NCI-ALMANAC dataset as the benchmark to evaluate the performance of the proposed method. The NCI-ALMANAC is a library of cancer cell lines maintained by the National Cancer Institute (NCI) [8]. The original NCI-ALMANAC datasets provide the anticancer drug information for 60 cell lines obtained from nine cancer types. In the experimental settings, the paper filtered out the dataset that only considered drugs with at least one target gene. Finally, the filtered dataset contains 130182 pairs of drug combinations.

The article "DCE-DForest: A Deep Forest Model for the Prediction of Anticancer Drug Combination Effects" was published in 2022. Journal: Comput Math Methods Med.

### 2.2. Pipeline of DeepDDS

DeepDDS (deep learning for drug-drug synergy prediction) is a deep learning model based on graph neural network and attention mechanism, which can learn drug characterization from chemical structure [6]. BERT model (Bidirectional Encoder Representations from Transformers) is a deep bidirectional language representation model based on transformer. Its essence is to construct a multilayer bidirectional encoder network using transformer structure, which has strong feature extraction ability. Inspired by DeepDDS model, BERT model and random forest (RF) regression algorithm can be used to predict the results of anticancer drugs. Thus, we propose a dynamic contrast-enhanced deep forest model (DCE-DForest) to predict the synergistic effect of drug combination. There are two components in the proposed DCE-DForest: (1) the pretrained drug BERT model to encode the drug based on the SMILES; (2) the synergistic effect (synergistic or antagonistic) will be predicted based on embedding vectors of drug and cell line by the deep forest method. The DCE-DForest learning framework is shown in Figure 1.

The drug embedding is obtained through pretrained drug BERT model. The embedding vectors of drug and cell line are concatenated to feed into the deep forest to predict the synergistic effect.

### 2.3. Drug Representation Based on Pretrained Drug BERT Model

The main idea in this paper is to apply deep learning methods to the SMILES string to learn meaningful patterns from the atoms and bonds. This knowledge should help create models that predict molecular properties from first principles and without explicitly encoding rules from chemistry. A variety of deep learning models have been proposed to represent the SMILES string. However, the vast chemical space together with the limited availability of labels makes supervised learning challenging, demanding learning a general-purpose molecular representation. Recently, pretrained transformer-based language models (PTLMs) on large unlabeled corpus have produced state-of-the-art results in many downstream natural language processing tasks. Inspired by this development, here the paper applied the pretrained drug BERT model to encode the drug SMILES [9].

Given a drug, let *M*_*s*_ = (m_1_, m_2_, ∙∙∙, m_l_) denote the SMILES, where *l* is the length of *M*_*s*_. The special [CLS] and [SEP] tokens were added to the *M*_*s*_ and fed into the pretrained BERT model to generate the drug representations. Subsequently, authors use the output of the last layer as the drug representation of [CLS] token to predict the synergistic effect of the drug combination [9].

The article "DCE-DForest: A Deep Forest Model for the Prediction of Anticancer Drug Combination Effects" was published in 2022. Journal: Comput Math Methods Med.

### 2.4. Deep Forest

The deep forest, also known as GCForest (multigrained cascade forest), is a novel deep learning method. Deep forest algorithm has constructed the deep learning mode of nonneural network structure for the first time and has become a research hotspot in the field of machine learning algorithm because of its excellent characteristics of nondifferential form-based learning device and no need of a large number of training data. Its main advantages are as follows: (1) it has good generalization performance when there are few training data; (2) the number of cascade layers is adjusted adaptively with the training process; (3) few superparameters and insensitive to the adjustment of super parameters; and (4) it has the structure of parallel processing.

As an alternative to deep neural networks, deep forest has been successfully applied to various applications in bioinformatics field, such as lncRNA-miRNA interaction [10], breast cancer subtype classification [11], and protein-protein interaction [12].

The gene expression profile is used to represent the cell line. All the NCI-ALMANAC dataset cell line features can be downloaded from CellMinerCDB [13]. Firstly, the feature vector obtained by the BERT model and the gene expression of cell lines is concatenated to feed into the deep forest to predict the synergistic effect. Secondly, DCE-DForest expands the first layer by training forests using the concatenated the feature vectors. In order to reduce the risk of overfitting, the class vectors output from each forest are generated by *k*-fold cross validation; that is, each instance will be treated as training data *k*-1 times, generate *k*-1 class vectors, and then calculate the mean value, concatenate them with the features in the raw features, and then take them as the input of the next layer. After the DCE-DForest being extended to the next layer, the performance of the DCE-DForest will be estimated on the validation set. If there is no significant performance gain, the training process will terminate. Thus, the DCE-DForest can determine the complexity of its model by properly terminating the training, which makes DCE-DForest suitable for different scale training data while not being limited to large-scale training data. Then, calculate the average of the probability of each category generated by all forests in the last layer. In the prediction process, the category with the maximum probability value is the final prediction result.

## 3. Results and Discussion

### 3.1. Evaluation Metrics

In this study, the NCI-ALMANAC dataset was randomly split into 80% training set and 20% test set and was repeated five times to evaluate the model performance. The following metrics are applied to evaluate the performance of DCE-DForest and other existing methods:

(1) $$\begin{array}{c} \text{Precision}=\frac{\text{TP}}{\text{TP}+\text{FP}} \end{array}$$

(2) $$\begin{array}{c} \text{Recall}=\frac{\text{TP}}{\text{TP}+\text{FN}} \end{array}$$

(3) $$\begin{array}{c} \text{Accuracy}=\frac{\text{TP}+\text{TN}}{\text{TP}+\text{FP}+\text{TN}+\text{FN}} \end{array}$$

(4) $$\begin{array}{c} F_{\beta }-\text{score}=\frac{\left(1+\beta^{2}\right)\times \text{Precision}\times \text{Recall}}{\beta^{2}\times \text{Precision}+\text{Recall}} \end{array}$$

where TP is true positive, FP is false positive, FN is false negative, and TN is true negative. Precision measures how accurate the model is in classifying the drug combination pairs as synergistic, and recall refers to the percentage of total synergistic drug combination pairs that were correctly classified. Accuracy (ACC) is a metric that describes the ratio between the correctly classified synergistic drug combination pairs and the total drug combination pairs in the dataset. *F*_*β*_ − score is a comprehensive metric that combines precision and recall. In the experiments, *β* is set to be 1 so as F_*β*_ − score is called F1-score. Besides, the paper also uses the area under ROC (receiver operating characteristic) curve and area under the PR (precision and recall) curve to measure model performance, called F1-score.

The article "DCE-DForest: A Deep Forest Model for the Prediction of Anticancer Drug Combination Effects" was published in 2022. Journal: Comput Math Methods Med.

### 3.2. Comparison of Drug BERT Embedding with the Traditional Drug Features

In this study, seven distinct traditional drug features (ECFP, LECFP, FCFP, Avalon, MACCS, HashTT, and RDKF) were used as the benchmark features in order to compare the BERT embedding for drug. The results are shown in Figure 2. As can be seen from Figure 2, the BERT embedding is superior to other drug features under the AUC (area under ROC curve) and AUPRC (area under precision recall curve) metrics. The reason is that the BERT has a more powerful embedding ability than the traditional drug features and can retain the important feature information of drug more completely.

### 3.3. Comparison of DCE-DForest with the State-of-the-Art Model

To evaluate the performance of DCE-DForest, DCE-DForest model is compared with some current state-of-the-art methods, including XGBOOST [14], logistic regression (LR) [15], DeepSynergy [2], and NN-XIA [3]. These models are excellent algorithms in the field of anticancer drug effect prediction in recent years. They have the advantages of wide application and high recognition.  Table 1 reports the performance of the compared methods with DCE-DForest method based on ACC, F1-score, recall, precision, AUC, and AUPRC. Under the operating environment of CPU Core i7 series, 64G memory, and Linux Ubuntu 20.04 LTS, the calculation results are shown in Table 1. As shown in Table 1, DCE-DForest achieved higher AUPRC than all other methods, and its performance measures of ACC, F1-score, recall, precision, and AUC reach 0.976, 0.334, 0.222, 0.676, and 0.921, respectively. Although XGBoost's performance is fairly good, it is still not as good as DCE-DForest. In terms of computational efficiency, the computing time of various algorithms is on the millisecond level, with little difference.

The article "DCE-DForest: A Deep Forest Model for the Prediction of Anticancer Drug Combination Effects" was published in 2022. Journal: Comput Math Methods Med.

The three deep learning-based methods, DCE-DForest, DeepSynergy, and NN-XIA, outperform the XGBoost and LR. The reason why deep learning methods are better than traditional machine learning method is that deep learning methods can extract effective abstract representations from the data. It is conceivable that with the accumulation of more and more data of drug combination, the gap between deep learning methods and traditional machine learning methods will become larger.

As for deep learning models, NN-XIA achieves the second-best prediction performances. The advantage of NN-XIA to obtain better performance than DeepSynergy is that it processes input features in different ways. The NN-XIA utilizes submodules to extract high-level abstract feature for the inputs, while DeepSynergy combines all types of input features and utilizes the feed-forward neural network to predict the drug combination effects. This also suggests that designing more sophisticated feature processing models may be more helpful to the prediction results.

## 4. Conclusions and Next Works

In this paper, a novel end-to-end deep learning method has been proposed to predict synergistic drug combinations. The pretrained drug BERT has been used to extract features from drug SMILES. Then, the synergistic effect of drug pairs is predicted by deep forest based on the concatenated features of drug and cell lines. Experimental evaluations show that DCE-DForest model performs significantly better than the traditional drug features and other competitive methods. Based on the experimental results, a conclusion is drawn that DCE-DForest can be effectively applied to predict synergistic drug combinations.

We could investigate the impact of the hyperparameters on explanations in future work, such as measuring the numbers of explanations, the distribution of their sizes, and their diversity in terms of features occurring in explanations; the number of trees especially in DCE-DForest was tuned to ensure that the accuracy of DCE-DForest model is good enough.

The article "DCE-DForest: A Deep Forest Model for the Prediction of Anticancer Drug Combination Effects" was published in 2022. Journal: Comput Math Methods Med.

## Figures and Tables

**Figure 1:** The pipeline of DCE-DForest learning framework.

**Figure 2:** Plot of AUC and AUPRC for different drug features.

**Table 1:** Model prediction performance comparison result.

Model	ACC	F1-score	Recall	Precision	AUC	AUPRC
XGBOOST	0.976	0.274	0.172	0.663	0.888	0.361
LR	0.972	0.06	0.031	0.487	0.853	0.203
DeepSynergy	0.975	0.311	0.207	0.631	0.907	0.382
NN-XIA	0.976	0.314	0.208	0.682	0.913	0.422
DCE-DForest	0.976	0.334	0.222	0.676	0.921	0.428

## Data Availability

The NCI-ALMANAC data used to support the findings of this study are available from NCIDTPdata/NCI-ALMANAC.
